The article "Career Development Anxiety and Mental Health Regulation of University Music Teachers" was published in 2022. Journal: J Healthc Eng.

# Career Development Anxiety and Mental Health Regulation of University Music Teachers

**DOI:** 10.1155/2022/9091795

**Published:** 2022-02-28

**Authors:** Hua Yan

**Affiliations:** School of Art, Zhejiang Yuexiu University, Shaoxing 312000, China

## Abstract

Mental health essentially refers to a state of mind. It means that an individual can keep a good or normal state in behavior. It is not only related to the overall development of the individual body and mind but also affects the construction of university teachers. This paper mainly studies the career development anxiety of music teachers in colleges and universities in China, analyzes its causes, and puts forward corresponding countermeasures and suggestions to alleviate the pressure and promote the physical and mental harmony of music teachers and the common growth of a good social atmosphere. The purpose is to help music teachers in colleges and universities better manage their mental health. This paper collects the data of occupational stress and mental health of 164 music teachers in many colleges and universities through the method of a questionnaire survey and processes the data with the analysis formula of sample variance and standard deviation. The analysis shows that a considerable number of the respondents have career development anxiety.

## 1. Introduction

The inequality between social progress and the reform of professional titles in higher education has always been a huge stone in the hearts of all teachers. In the past, we have always unilaterally emphasized that teachers should have the spirit of dedication but ignored the pressure they bear as a special social group and the reasonable demands for normal career development [1, 2].

After entering the new century, the research on the occupational stress of primary and secondary school teachers in China is gradually deepening, but the research on the occupational stress of college teachers has not attracted enough attention. Although university teachers do not face the pressure of students' entrance examinations, the students they face have more mature personalities, and the form of classroom teaching is more open. Students often put forward some problems that teachers cannot explain in class. All of these lead to the fact that college teachers are also suffering from unimaginable social and psychological pressure [3].

According to the survey data, more than 72.3% of young college teachers in China think that their work and academic research pressure is too high, which makes them often fall into more serious mental health problems [4]. In addition, many colleges and universities in our country adopt the incentive policy of “go or not”, which makes young teachers in colleges and universities who are in deep trouble feel more confused about their career prospects.

A work stress survey of young university teachers found that the mental health of young university teachers has deteriorated year by year. Especially in recent years, the impact of pressure on young university teachers, such as low wages, difficulty in buying a house, and difficulty in promotion, has gradually increased. The state of mental health is getting more and more severe, as shown in Figure 1.

It can be seen from Figure 1 that the mental health index of young teachers in colleges and universities decreases year by year as the years increase. Taking 2015 as the best starting point for health, by 2021, the average health index has dropped by 30%. It can be seen that the mental health of young music teachers in colleges and universities is deteriorating rapidly.

The psychological state has an important influence on an individual's life and work. The influence of teachers' mental health on the sustainable development of education cannot be ignored [5, 6]. To pay attention to their mental health, and to achieve positive intervention on their mental health by building a good career development space and strengthening psychological counseling is a necessary way to improve the working state of college teachers in China [6, 7]. The mental health of university teachers will not only affect their own work and study but also bring great differences to students' learning moods and even their cognition of the world. There is an obvious positive relationship between the two. College teachers with good mental health will make students feel more sunshine in their studies and life, and vice versa [8, 9]. In many cases, these two opposite learning emotions will accompany students throughout their lives. Human resource management in colleges and universities, as an important entry point to improving the professional development space of college teachers, should not only focus on the teaching work and academic achievements and other hard indicators, but also expand to include the guidance and intervention of teachers' mental health so as to create a more three-dimensional and comprehensive work system of teachers' mental health and help college teachers to work more actively and effectively and improving their healthy psychological state to carry out education and teaching work. [10, 11].

As a nonmusic college, music teachers are a relatively special group. They are more in line with the perceptual cognition of university teachers: brilliant and easy to work with. As a result, their career development anxiety is more easily ignored by society [12, 13]. Paying attention to the mental health regulation of this group not only helps to solve the mental health problems they are facing, but also has a very important reference value for the mental health regulation of the whole team of university teachers.

## 2. Professional Development Anxiety and Psychological Adjustment of College Music Teachers

### 2.1. Characteristics of the Professional Development of College Music Teachers

#### 2.1.1. Particularity of Music Teachers

Music teaching pays attention to aesthetics just like dance and art, and music learning is not a day's work. It requires years of learning. In addition, music learning is not only about professional knowledge, but more importantly, experience in life. The profession of a music teacher is different from other teachers, mainly in the following aspects.

First, after becoming a music teacher, you can combine your profession and expertise, find a suitable entry point, combine your expertise with teaching, and promote the continued development of music.

Second, there is a very close relationship between the professional development of music teachers and the school environment. These development environments mainly include the relationship between the internal environment and the external one [14, 15]. The internal environment mainly refers to people's innate sensitivity to music and various physiological conditions such as their voice, while the external environment mainly refers to people's in-depth research and pursuit of music.

Third, the professional development of music teachers has always been a straight line, and there are no other diversions. Despite this, music teachers also face all kinds of difficulties, but they still work hard to form their own unique teaching styles and models.

#### 2.1.2. Features of Professional Development of Music Teachers in Colleges and Universities

*Phased*. Music teachers are of different ages, and their development will also show different developmental characteristics. At different ages, the problems they face will be different. This is the stage. According to research, 25–60 years old can be called an adult stage. Music teachers between the ages of 25–35. They are young and energetic and have innovative ideas in music. At this time, they are faced with problems in career planning, life planning, and family formation, such as employment, studying abroad, falling in love, and getting married. Music teachers at the age of 35–50 have completed family formation-related issues and accumulated a lot of social experience. They are calm and efficient in their work, and their bodies and spirits are at the peak of activeness. Music teachers at the age of 50–60 may not be as good as the previous two stages, but they have profound professional knowledge, the richest teaching experience, and the highest level of scientific research. According to the statistical results of university research institutions, it is found that the occupational anxiety of college music teachers will increase first and then decrease with age. The specific situation of anxiety is shown in Figure 2.

It can be seen from Figure 2 that the occupational anxiety value of young college music teachers between the ages of 30 and 35 reaches the highest level, and with the increase in age, the occupational anxiety value of college music teachers gradually decreases, reaching the lowest point at the age of 60.

*Dynamic*. Music teachers are also a group of society [16]. They are also in a social environment. Their career development cannot be separated from the influence of the environment, and this influence is also mutual. The activities of music teachers will also have an impact on the environment [17, 18]. The stages mentioned in the previous article also show that the professional development of music teachers is dynamic and constantly changing, which only shows that different ages lead to different environments, which will have an impact on the professional development of music teachers. In addition, when college music teachers leave the university campus, there are not many career choices. Maybe a certain institution becomes a training teacher. Therefore, it is best for college music teachers not to leave the university campus to develop independently.

*Comprehensive*. Comprehensiveness means that in the process of professional development, college music teachers must not only have their own unique professional style and authority but also have the knowledge and teaching management capabilities related to other disciplines [19]. As a teacher, they must have at least pedagogy-related knowledge, be good at getting along with students, discover the characteristics of students, and should know how to guide students with different physical conditions to guide their music professional learning. In addition, music teachers must have strong music creation abilities and practical abilities, and constantly improve their level of professional knowledge and innovative teaching methods.

### 2.2. Performance of College Music Teachers' Occupational Anxiety

Through the analysis of data from different institutions, it is shown that the performance of occupational anxiety of music teachers in colleges and universities is mainly divided into four types. Among them, the degree of influence of different types of anxiety on the teachers' mental health index is shown in Figure 3.

It can be seen from Figure 3 that the performance of college music teachers' occupational anxiety is mainly divided into four types. Among them, grumpy type anxiety has a high impact on teachers' mental health index, reaching 31.58%, while suspicious and uneasy types of anxiety have the lowest impact on teachers' mental health index, at only 19.3%.

It can be seen from Figure 3 that all kinds of anxiety will adversely affect the mental health of college music teachers. The specific types of anxiety involved are as follows.

*Emotional Pessimism*. When music teachers are dissatisfied with their current work, they will be pessimistic. They often feel exhausted, and it is difficult to show a happy expression about something. Most of the time, they see the negative side of things first. The time spent alone is prolonged, and interpersonal communication is extremely lacking. Too worried about the future and then become gloomy, even during the teaching period, they would not shy away from it. Over time, this emotion will infect students and other teachers.

*Grumpy*. Music is inherently unique in art, and music teachers also have very obvious personal characteristics. When society, parents, and schools intervene in their teaching too much, they feel that they cannot concentrate on studying music or even become secular. Sometimes they will become very irritable. In teaching, they will be more demanding on students. They will be less tolerant of students who make mistakes. They often become inexplicably angry. They will be self-centered, not cooperate, and not listen to other people's advice, which makes the job impossible. To proceed in an orderly manner, seriously interfering with teaching work.

*Suspicious and Uneasy*. When teachers are hit, they are prone to self-doubt or feel that others are deliberately targeting themselves, and when they start to think about themselves and their insecurity, the whole person's defensiveness becomes heavier and he is unwilling to communicate with others. In the long run, insomnia and overreaction are prone to occur, which seriously affects normal teaching and life, creates greater obstacles to professional development, and will aggravate teachers' professional anxiety.

*Nervousness*. Nervousness manifests itself as being overly entangled in something, speculating on the adverse consequences of the event, fear of making mistakes, excessive worry about the past and future, fear of losing face, always being cautious, and pursuing too much perfection.

### 2.3. Psychological Adjustment Countermeasures of College Music Teachers

#### 2.3.1. Create an Environment Conducive to the Mental Health of Teachers

Teachers bear the heavy responsibility of preaching and receiving jobs, and their mental health has a huge impact on society. Local governments should earnestly safeguard the rights and interests of teachers. To solve the psychological problems of music in colleges and universities, it is necessary to find the source of the problem, counter the medicine, create an easy-to-teach working environment for college music teachers, improve the salary and social status of college music teachers, and conduct regular mental health education for college music teachers. Practical actions should be taken to solve the difficulties that teachers encounter in life and work.

#### 2.3.2. Adhering to the People-Oriented Education Management Method

In terms of adjusting the psychological state of music teachers in colleges and universities, it is necessary to optimize management methods and management models through local colleges and universities, always adhering to the people-oriented management philosophy, attaching great importance to the mental health of teachers, and carry out relevant training activities on a regular basis. In addition, formulate more scientific and reasonable teacher assessment standards and prohibit the establishment of standards that ignore reality. When recruiting teachers, we should also pay attention to the mental health of teachers and create a team of teachers with a good atmosphere. Formulate incentive policies that take into account teachers' contributions and achievements at work, and at the same time strictly require teachers' ethics and morality. They must also be rigorous in academic research to avoid mental health problems caused by bad academic habits. Reasonable control of the working hours, advocating the combination of work and rest, and holding faculty sports games or art evenings to provide teachers with more opportunities to show themselves.

#### 2.3.3. Improving the Psychological Quality of Teachers Themselves

At the same time, teachers should also understand that their responsibilities are heavy, introspect in time, and improve their level of professional knowledge for teaching and ideological and moral cultivation. At the same time, they must also understand that they are the object of the students' respect, and they must be able to convey positive energy to the students rather than vent their negative emotions on the students. Survival of the fittest has always been the rule of the world. If they want to develop better, they must improve their overall quality, including psychological quality, in order to strengthen their professional knowledge. This requires teachers to learn to control their emotions and handle things calmly. To have a clear understanding of oneself, they should face up to one's own shortcomings and deficiencies, accept different opinions from the outside world, establish good interpersonal relationships with colleagues, treat students equally, and learn to tolerate others.

When the teachers realize that they are feeling irritable and stressed, they must learn to find solutions. Schools and students are the objects teachers can seek for help. Teachers should not feel ashamed to speak out when they have psychological problems. They should open their hearts to communicate with others. Closing themselves will only make the results worse and worse. They should learn to advance with the times, constantly improve themselves, and adapt to the surrounding environment. Actively participating in school activities, having the courage to show oneself, not caring too much about gains and losses, seeing the false name, teaching and educating people, and academic research are what teachers should care most about.

#### 2.3.4. Developing Good Living Habits

Healthy living habits have always been an important prerequisite for physical and mental health. Music teachers or other teachers in colleges and universities will not change to tie themselves to research and professional titles. They must always be happy so that they can work in order to achieve the effect of getting twice the result with half the effort.

1. Good sleeping habits can help music teachers in colleges and universities to be energetic and comfortable at work, reducing the intake of unhealthy stimuli such as coffee, tea, tobacco, and alcohol before going to bed, and forming and creating a suitable sleeping environment will also help;
2. Scientific eating habits and scientific diets provide energy support for teachers to engage in heavy mental work. The specific requirements are timing, quantitative, reasonable collocation, no partial eclipse, and attention to food hygiene;
3. Appropriate leisure activities can relax teachers' bodies and minds, satisfy hobbies, and experience the function of self-growth. Occasionally, a movie or drama, a walk in the park, a visit to a painting exhibition or a museum, etc., will make them feel physically and mentally happy and stress relieved;
4. Reasonable physical exercise can strengthen the body, beautify the image, and at the same time help increase teachers' self-confidence, self-esteem, self-control, and self-satisfaction, and more importantly, relieve work and psychological pressure. Physical exercise is the best way to get rid of negative emotions and prevent depression, anxiety, and worries.

## 3. Investigation and Experiment on the Stress and Mental Health of Music Teachers in Colleges and Universities

### 3.1. Experimental Content

Music teachers are a group of teachers with distinctive personalities, but they are also prone to psychological problems. This experiment mainly selected 4 colleges and universities in the province as the experimental site, took the music teachers of these 4 colleges and universities as the research objects and investigated their occupational stress and mental health problems. This experiment adopts the experimental method of a questionnaire survey. A total of 175 questionnaires were distributed to music teachers in these 4 universities, and 164 valid questionnaires were returned. The survey tool used the SCL-90 symptom self-rating scale.

### 3.2. Experimental Process

The survey content was determined and the questionnaire questions were set up. The questionnaire is completed in accordance with the design criteria of the questionnaire. The survey subjects are communicated with before the survey, and after an agreement is made, the survey staff will hand out the questionnaire and the music teacher will fill it out on the spot. It took one week from the issuance of the questionnaire to the collection of the questionnaire. After that, the collected questionnaires were sorted out and the data was collected. The formula used in the data processing stage is as follows:

(1) $$\begin{array}{c} \text{Sample variance formula}:s^{2}=\frac{\sum_{i=1}^{n}{\left(x_{i}-x\right)}^{2}}{n-1},\\ \text{Sample standard deviation formula}:s=\sqrt{s^{2}}=\sqrt{\frac{\sum_{i=1}^{n}{\left(x_{i}-x\right)}^{2}}{n-1}}. \end{array}$$

## 4. Survey Results of the Professional Pressure and Mental Health of College Music Teachers

### 4.1. Survey on the Severity of Occupational Anxiety and Mental Health

The relevant standards of the SCL-90 symptom self-rating scale have stated that the factor score is greater than or equal to 2 as a mild symptom response. When the molecular factor is greater than or equal to 3, it means that the survey subject has a moderate or higher symptom response.  Figure 4 shows the statistics based on the relevant standards of SCL-90:

Figure 4 shows that college music teachers may have various possible problems, including psychological problems such as somatization force, Interpersonal sensitivity, depression, anxiety, hostility, terror, paranoid, and psychotic.

Among the 164-people surveyed, 99 people had mild symptoms and 65 people had moderate or above symptoms. From this point of view, the professional pressure on music teachers in colleges and universities in the province is relatively high, and their mental health problems have gradually become prominent.

It can be seen from Figure 4 that among the mild symptom responses, the most prominent is the interpersonal relationship. The number is 90, which is more than half of the sample. Secondly, self-anxiety and physical factors are also compared among them.

Among the above-moderate reaction symptoms, self-anxiety is also the most prominent. The number of people with this factor is 25.

Through further analysis of the results of the questionnaire, the anxiety index is defined in the interval (0, 1), and then the value of a single survey result is quantified, compared with the quantified value of the entire survey sample, and the value of each survey sample is calculated. Anxiety values and the corresponding extreme values, average values, and anxiety states are analyzed and the specific display is shown in Table 1.

It can be seen from Table 1 that the lightest symptom of occupational anxiety for music teachers in colleges and universities is 0.18, and the worst symptom is 0.92. The average of the occupational anxiety symptoms of music teachers in colleges and universities is 0.72. Through the analysis of the mean value, it can be seen that the overall anxiety level of the 164 teachers in this survey is at an upper-middle level.

### 4.2. Attitudes of Music Teachers to Occupational Anxiety and Mental Health Problems

Figure 5 shows the survey results on the attitudes of music teachers to occupational anxiety and mental health problems. The figure shows that 68% of teachers adopt a positive and optimistic approach, and 16% of teachers feel that there is no need to pay attention and just let it develop. 6% of the teachers were unaware of the problem, and 10% of the teachers took other methods to solve it.

## 5. Conclusion

Music teachers are the most important team force to support music aesthetic education in colleges and universities. Their mental health will undoubtedly have a subtle impact on college students' studies and lives. Taking the opportunity of career development and reform, we must pay attention to the key topics of professional improvement and mental health adjustment of music teachers in colleges and universities. Teachers are humans too. Since they are humans, there are problems of survival and development. If these problems cannot be resolved in a timely and effective manner, psychological diseases may result. Patients suffering from severe psychological diseases may pose a certain threat to their family, society, and school. Music teachers in colleges and universities should pay attention to the improvement of their theoretical knowledge of mental health, and school management departments and society should also pay attention to the mental health of college music teachers, organizing various activities to improve teachers' mental health levels, promoting teachers' physical and mental health, and school education in a harmonious development.

Colleges and universities should create an environment conducive to the mental health of teachers and adhere to a people-oriented education management method. Music teachers in colleges and universities should also take the initiative to improve their own psychological quality and develop good living habits in peacetime. In short, the adjustment of the mental health of college music teachers requires the joint efforts of colleges and teachers. Only by maintaining a good mental state can college music teachers have better professional development.

## Figures and Tables

**Figure 1:** The mental health of young teachers in colleges and universities.

**Figure 2:** The changing trend of anxiety of college music teachers with increasing age.

**Figure 3:** The degree of influence of different types of anxiety on teachers' mental health.

**Figure 4:** Distribution map of problem severity.

**Figure 5:** Music teachers' attitudes towards occupational anxiety and mental health problems.

**Table 1:** Occupational anxiety index of college music teachers.

Number of respondents	Mean anxiety	Maximum anxiety	Anxiety minimal	General anxiety state
164	0.72	0.92	0.18	Middle

## Data Availability

The datasets used and/or analyzed during the current study are available from the corresponding author on reasonable request.
